RETRACTED

# Economic Growth Effect of Public Health Investment and Its Impact on Living Environment

**DOI:** 10.1155/2022/2192255

**Published:** 2022-05-26

**Authors:** Jinglei Meng

**Affiliations:** Department of Financial Management, School of Economics and Management, Harbin University, Heilongjiang, Harbin, China

## Abstract

Based on the concern of Chinese residents for health and the improvement of related service demand, this paper studies the economic growth effect of public health investment and its impact on living environment by analyzing the determination coefficient estimated by Spearman and nonlinear curve. The results show that the impact of increasing government financial public health investment on regional economic growth rate is not only related to regional economic aggregate and development level, but also related to regional education level and regional publicity level in logical analysis. The improvement of residents' living environment brought by public infrastructure investment can effectively stimulate residents' concept of health consumption and then make the economy of nonpublic health undertakings achieve a higher growth rate. The economic growth rate brought by nonpublic health undertakings is also an important component of the local economic growth rate. It can be seen that strengthening the infrastructure construction of urban living environment can not only improve the overall living environment quality of the city, but also promote the development of the city and the development speed of the city.

## 1. Introduction

With the improvement of China's economic level, the living materials of residents have been greatly enriched. With this, residents pay more and more attention to health, and their demand for health-related services has gradually increased. After a highly civilized society, health not only refers to physical diseases and the performance of qualitative strength, but also includes psychology and the ability to adapt to society. Public health investment is the economic cost of counseling to maintain residents' physical and mental health and social adaptability. Health investment is a project beneficial to the public. It is mainly to enable the public to have a healthy physical and mental health and a better and happy life, especially after social progress, and after people's demand for spirit and material increases, people's life pressure increases. Subhealth and psychological problems perplex the young generation. It leads to some negative phenomena in the process of work, life, and study of the young generation, which affects the benign development of the social environment.

People or animals living on the Earth depend on the natural environment to survive (Jing Zhongping (2021)). The living environment is closely related to the living conditions of people or animals. Especially with the progress of science and technology, in order to pursue a more comfortable living environment, people use artificial intelligence to intervene in the surrounding environment and create a good living environment by adjusting the temperature, lighting, and ventilation of the environment. It is beneficial to improve the milk production efficiency of dairy cows [1]. Due to geographical and cultural differences, people's living habits and diet are different, and the personalities of people in the South and the North are quite different (Zhang Jiawei (2021)). When there are relevant data sheets, the probability of cardiovascular disease in patients in northern China is higher than that in the south. However, there is no targeted solution for this phenomenon, which can only be attributed to the impact of the living environment on people's habits, resulting in some negative effects [2]. After the improvement of living standards, people's material pursuit will shift to spiritual satisfaction, and they will also focus on their own health management (Qian Xiangli (2021)). Through the analysis of the relationship between public health investment and personal health management investment in Jiangsu Province, it is found that public health investment will positively affect the investment in personal health management, while the investment in personal health management has little impact on public health investment. Through the in-depth study of the relationship between them, it is helpful for the state to adopt corresponding strategies for health investment [3]. Zhang Fen (2017) compared the impact of public health investment and private health investment on economic growth. The results show that health investment can significantly promote economic growth, but there is a crowding out effect between them, and the proportion of public health investment varies according to different regions [4].

RETRACTED

Everyone needs a healthy physique, so everyone needs to participate in health investment, and building a healthy country needs the comprehensive quality of national health. At the same time, individuals and families need health protection to realize a happy life. Therefore, health is not only a social responsibility, but also an individual's behavior. This study mainly starts from the regional direction to study the effect of public health investment on economic growth and the living environment.

## 2. Related Concepts and Literature Review

### 2.1. Public Health and Public Health Investment

The public health of residents plays a vital role in the development and progress of society. Only when the personal health level meets the requirements can we wholeheartedly provide assistance for the development of society. This also affects the intensity of public health investment. Public health investment is mainly aimed at the investment of the state, the government, and social public departments in social medical care that can ensure the health of residents. Public health investment has a positive impact and role in promoting the development of national health and medical and health undertakings, improving the overall health quality of citizens and promoting the harmonious development of society. Yao Yanan's research (2018) shows that public health is closely related to the development of urban green space, so it is necessary to explore and study the correlation between them [5], and green space can also be designed according to the influence mechanism, so as to promote the development of public health. Li Jingwei (2020) studied the correlation between land use and public health and systematically combed the impact of land use on public health through literature analysis [6]. It can also be proved that the use of land can have an impact on the surrounding environmental quality, thus affecting public health.

For personal health, the base of public health is large, and public health is an important part of human capital, and public health investment is an effective way to improve public health. With the attention of society and individuals on public health, the intensity of public health investment will increase [7]. It is emphasized that the public health system should adapt to and promote the construction of economic, political, cultural, social, and ecological civilization of the country (region) where it is located Li Chengyue et al. (2021) [8]. Public health investment can help people obtain the means of living, medical and health services, and resources and time needed for good health. Establishing and improving the basic social health security mechanism is the embodiment of the good development of the country and society, as well as the embodiment of political civilization, material civilization, and spiritual civilization.

### 2.2. Healthy Economy and Regional Economy

Through the statistical analysis of the national, local, financial, medical, and health expenditure, the whole country is divided into four regions according to the orientation: the east, the middle, the southwest, and the northeast, and the health economy and regional economy of these four regions are analyzed, respectively. The proportion of public health investment in the four regions is in the southwest from large to small [9]. East, central, and northeast: There are two reasons for the differences: one is the inclination and implementation of the government's policies in various regions; second, the economic development of the region itself is different. The geographical location of the eastern region is dominant, and the surrounding resources and technology will drive the local economic development. The data in Table 1 below show the financial public health expenditure in different regions from 2014 to 2019 according to the National Bureau of Statistics.

RETRACTED

It can be seen from the data in Table 1 that the financial medical and health expenditure in all regions increases year by year, but the growth trend is different. The state's expenditure on medical and health care has also improved residents' attention to their own health awareness. The better the health status of residents, the better their living conditions, and living standards will be further improved. Therefore, while effectively improving the health level of residents, the regional economy will also be vigorously developed, providing a strong guarantee for people's life.

### 2.3. Living Environment and Quality of Life

People's living environment will not only have an impact on the local economy, but also have the most direct impact on people's pursuit of quality of life. Having a good living environment can enhance residents' love for life and will not muddle along, which will indirectly improve residents' quality of life. Qiu Jiahong (2021) studied the living environment of the mixing town and found that the natural combination of “arbor, shrub, and grass” is reasonable, so the living environment is better [10]. The living environment also plays a vital role in education. Wang Tingyu (2020) showed the importance of the living environment for early childhood education. A good living environment provides possibilities for early childhood education and also affects the educational content and quality because life materials are the best educational content [11].

## 3. Correlation Analysis of Regional Characteristic Economy

### 3.1. Spearman Correlation

Spearman correlation algorithm:

(1) $$\begin{array}{c} \rho_{s}=\frac{\sum_{i=1}^{N}\left(R_{i}-\bar{R}\right)\left(S_{i}-\bar{S}\right)}{{\left[\sum_{i=1}^{N}{\left(R_{i}-\bar{R}\right)}^{2}\sum_{i=1}^{N}{\left(S_{I}-\bar{S}\right)}^{2}\right]}^{1/2}}. \end{array}$$

Here, *R*_*i*_ and *S*_*i*_ are the grades of the observed values, respectively; $\bar{R}$ and $\bar{S}$ are the average grades of variables x and y, respectively; and N is the total number of observations.

### 3.2. Determination Coefficient of Curve Estimation

Coefficient of determination R2:

(2) $$\begin{array}{c} R^{2}=\frac{\sum_{i}\left(x_{i}-\bar{x}\right)}{\sum_{i}\left(x_{i}-{\bar{x}}_{i}\right)},\;\bar{x}=\frac{1}{n}\sum_{i=1}^{n}x_{i}. \end{array}$$

Here, $\bar{x}$ is to investigate the arithmetic mean of sample sequence ${\tilde{x}}_{i}$ is the ith input value in the sequence and *n* is the number of investigation samples.

RETRACTED

### 3.3. Data Sources

Six cities are selected in the eastern region, including Xuzhou, Wuxi, and Changzhou in Jiangsu, Ningbo and Haining in Zhejiang, and Xiamen in Fujian. Six cities are selected in the central region, including Nanyang, Xuchang and Pingdingshan in Henan, Xiangfan and Huanggang in Hubei, and Yuncheng in Shanxi. Six cities are selected in Southwest China, including Kunming, Tengchong, and Pu'er in Yunnan, Baise, Beihai, and Liuzhou in Guangxi. Six cities were selected in Northeast China, including Anshan and Dandong in Liaoning, Tonghua and Baicheng in Jilin, and Hegang and Mudanjiang in Heilongjiang. The selection range of cities excludes provincial capital cities and other subprovincial cities, and the urban data are closer to the regional median. The specific data come from the provincial and municipal statistical yearbook data, government report data, Industry Association Statistics, etc.

## 4. Correlation between Economic Growth and Health Investment

In this model, the proportion of public health investment and residents' personal health consumption are used as the correlation coefficient of health investment. Among them, the proportion of public health investment refers to the proportion of the investment of finance, SASAC, and nonpublic investors in hospitals, health service places, and urban health facilities in the total investment of the city in the current year. The proportion of residents' personal health consumption refers to the proportion of health-related consumption in residents' disposable income, including but not limited to health examination, nutrition and health care, health consultation, and other fields. The proportion of government public health investment in total fiscal revenue is selected as the independent variable data in the model. Through statistical data analysis, it can be seen that the data of Southwest China are higher than those of other regions, and the economy of central China and Northeast China is also lower than that of eastern China. Therefore, increasing regional public health investment plays a good role in promoting local economic development.

Firstly, the curve estimation calculation of 11 linear and nonlinear functions is performed for the above data, and the highest R2 value in all functions is selected as the regression determination coefficient. Spearman correlation analysis is performed for two independent variables (the proportion of public health investment and the proportion of residents' personal health consumption) and one dependent variable (the year-on-year growth rate of regional economy), and the highest R2 value is selected *ρ* Value as the result of correlation analysis. The results obtained by the above statistical methods are shown in Table 2.

RETRACTED

In Table 2, it was found that the determination coefficient of all four groups of cities was *R*^2^ > 0.800, *P* < 0.01. The correlation results of 0.900, *P* < 0.01, show that the data of four groups of cities have significant correlation and coupling. We have to investigate the distribution law of two independent variables (the proportion of public health investment and the proportion of residents' personal health consumption), respectively, perform data visualization, and get Figures 1 and 2.

In Figure 1, the data expression of Southwest China is significantly higher than that of other regions. Only from the analysis of these data, the data sensitivity of economically relatively backward regions is higher, but the economy of central and Northeast China is also lower than that of eastern regions, and its data expression is lower than that of eastern regions. Therefore, the impact of increasing government financial public health investment on the regional economic growth rate is not only related to the regional economic aggregate and development level, but also related to the regional education level and regional publicity level in terms of logical analysis. The two data in Figure 1 are expressed as follows: (1) The economic development power of Southwest China is more sensitive to regional public health investment. (2) Increasing regional public health investment shows an upward trend in all four groups of cities; that is, increasing regional public health investment in any city can promote local economic development.

In Figure 2, the sensitivity of data in Southwest China is still the highest, followed by the eastern region, northeast region, and central region. The data expression is basically consistent with the data expression in Figure 1 given above. It can be considered that in the investment consumption, “two carriages” theory, the impact logic of personal health consumption, and public health investment on regional economy are completely consistent. Residents' attention to health investment can improve people's ability to resist diseases and promote the benign interaction among individuals, society, and economy. A healthy labor force is promoted by health investment, so as to better promote economic growth.

RETRACTED

## 5. Correlation between Living Environment and Health Investment

In the previous paper, two independent variables were used to conduct correlation analysis on the year-on-year growth of regional economy. The model goes further and restricts the urban living environment with public infrastructure investment (including but not limited to public health investment), that is, assuming that the living environment of urban residents with better urban infrastructure is better, two dependent variables are set in the model, which are the proportion of residents' health consumption and the economic growth rate brought by health investment of nonpublic economy. For the above data, we need to expand the curve estimation algorithm based on 11 curve functions, take the maximum determination coefficient R2, and expand Spearman correlation analysis to take the maximum *ρ*. The analysis results are shown in Table 3.

In Table 3, among all four groups of cities, the eastern city has the highest R2 value, but the northeast city has the Spearman correlation *ρ*; that is, the data expression of the four groups of cities is more similar. All four groups of cities had the result of *R*2 > 0.800, *P* < 0.01*ρ*>. The correlation results of 0.900, *P* < 0.01, show that the data of four groups of cities have significant correlation and coupling. Two dependent variables (the proportion of residents' health consumption and the economic growth rate brought by health undertakings invested by nonpublic economy) were investigated, respectively, and the data visual analysis was carried out. The analysis results are shown in Figures 3 and 4.

In Figure 3, in terms of data sensitivity, the eastern region is the highest, followed by the northeast, and central and southwest regions. In the current situation investigation, the distribution law of the curve is related to the integrity of the previous urban infrastructure. That is, cities with a higher degree of infrastructure completion continue to increase urban infrastructure investment, which will give greater impetus to residents' health consumption. At the same time, when the infrastructure investment of the four groups of cities accounts for more than 10% of the total financial expenditure, the proportion of residents' health consumption will have a steep rising edge, which is more significant in the data expression of eastern cities. That is, from the philosophical theory of qualitative change caused by quantitative change, the proportion of urban public infrastructure investment should reach more than 10%, so as to effectively stimulate residents' healthy consumption and achieve higher investment efficiency.

RETRACTED

In Figure 4, in terms of data sensitivity, the eastern region is the highest, the central region is the second, the northeast and southwest regions have the lowest data expression, and the curve trend is almost the same. This data rule is basically consistent with the data rule of public infrastructure investment and residents' health consumption rate in Figure 3. Through the joint observation of the data in Figures 3 and 4, we can get the following data characteristics: ① the improvement of residents' living environment brought by public infrastructure investment can effectively stimulate residents' concept of health consumption, so as to achieve a higher growth rate of nonpublic health industry economy; ② the economic growth rate brought by nonpublic health undertakings is also an important component of the local economic growth rate. Relevant studies show that increasing the infrastructure construction of the urban living environment is also of positive significance to the growth rate of other economic forms.

## 6. Strategies and Suggestions for Improving Residents' Living Environment

### 6.1. Cities Should Appropriately Strengthen Constructive Investment in Public Health

In the four groups of 24 cities involved in the study, increasing the amount of financial investment in public health can effectively stimulate the concept of health consumption of local residents, healthy individuals improve the level of healthy labor force, improve the employment opportunities of workers, and realize the income of their health investment, so as to further stimulate the growth of local economy. It can be considered that any city should focus on public health investment in infrastructure investment. However, in the investment of urban infrastructure, we should not be too inclined to the investment in the field of public health. In the above research, improving the level of urban public infrastructure can also achieve the corresponding pulling effect. If we unilaterally strengthen the investment in public construction in the field of health, it will directly affect other urban public functions, such as urban public transport, municipal roads, municipal water supply, and drainage. That is, a certain proportion of urban infrastructure investment in public construction in the field of health should be maintained to ensure that the urban environment is scientifically optimized [12].

### 6.2. Different Cities Have Different Economic Sensitivities to Investment in Public Health

The previous public infrastructure construction of different cities is different. The urban construction in the more developed areas in the East is relatively perfect, and its data sensitivity is stronger. The urban construction in other areas is relatively backward, and its data sensitivity is slightly lower [13]. Therefore, when cities carry out infrastructure investment in the field of public health, they should take into account the development status of the city itself. Areas with relatively backward urban infrastructure construction should first carry out more comprehensive urban infrastructure planning and investment and take the lead in improving the quality of the urban living environment, while relatively developed areas can directly increase public health investment, so as to stimulate a higher speed of urban development.

RETRACTED

## Figures and Tables

**Figure 1:** Relationship curve between the proportion of public health investment and the year-on-year growth rate of regional economy.

**Figure 2:** Relationship curve between the proportion of personal health consumption and the year-on-year growth rate of regional economy.

**Figure 3:** Correlation curve between public infrastructure investment and residents' health consumption rate.

**Figure 4:** Correlation curve between public infrastructure investment and the growth rate of nonpublic health undertakings.

**Table 1:** Financial health expenditure in different regions of the country.

Region	2014	2015	2016	2017	2018	2019
Whole country	10086.56	11868.69	13067.61	14343.05	15412.93	16417.6
East	3953.71	4610.42	5191.12	5685.58	6194.64	6691.63
Central section	2434.06	2901.83	3132.88	3449	3703.35	3935.21
Southwest	2983.43	3554.71	3882.12	4295.45	4582.1	4830.11
Northeast	715.36	801.73	861.49	913.02	932.84	960.65

Data source: annual data of the National Bureau of Statistics from 2014 to 2019.

**Table 2:** Correlation analysis results of original data of four groups of cities (economic growth and health investment).

Grouping	Coefficient of determination		Relevance	
	R^2^	*P*	*ρ*	*P*
East	0.905	0.006	0.913	0.005
Central section	0.867	0.005	0.924	0.006
Southwest	0.835	0.007	0.905	0.005
Northeast	0.855	0.004	0.915	0.007

**Table 3:** Correlation analysis results of original data of four groups of cities (living environment and health investment).

Grouping	Coefficient of determination		Relevance	
	R^2^	*P*	*ρ*	*P*
East	0.913	0.006	0.927	0.004
Central section	0.824	0.008	0.914	0.006
Southwest	0.847	0.007	0.892	0.005
Northeast	0.875	0.004	0.935	0.004

## Data Availability

The data underlying the results presented in the study are available within the manuscript.
